The article "Simplified method to perform CLARITY imaging" was published in 2014. Journal: Mol Neurodegener.

# Simplified method to perform CLARITY imaging

**DOI:** 10.1186/1750-1326-9-19

**Published:** 2014-05-26

**Authors:** Ekaterina Poguzhelskaya, Dmitry Artamonov, Anastasia Bolshakova, Olga Vlasova, Ilya Bezprozvanny

**Affiliations:** 1 Department of Medical Physics, St.Petersburg State Polytechnical University, St Petersburg 195251, Russia; 2 Laboratory of Molecular Neurodegeneration, St.Petersburg State Polytechnical University, St Petersburg 195251, Russia; 3 Department of Physiology, University of Texas Southwestern Medical Center at Dallas, Dallas, TX, USA

**Keywords:** CLARITY, See deep brain, Neuronal structure, 3D brain tissue reconstruction, Neuroimaging, Confocal, Two-photon

## Abstract

**Background:**

Imaging methods are used widely to understand structure of brain and other biological objects. However, sample penetration by light microscopy is limited due to light scattering by the tissue. A number of methods have been recently developed to solve this problem. In one approach (SeeDB) simple procedure for clarifying brain samples for imaging was described. However, this method is not compatible with immunostaining approach as SeeDB-prepared tissue is not permeable to the antibodies. Another technique for clearing brain tissue (CLARITY) was optimized for immunochemistry, but this method technically much more demanding than SeeDB.

**Results:**

Here we report optimized protocol for imaging of brain samples (CLARITY2). We have simplified and shortened the original protocol. Following hydrogel fixation, we cut brain tissue to 1–1.5 mm thick coronal slices. This additional step enabled us to accelerate and simplify clearing, staining and imaging steps when compared to the original protocol. We validated the modified protocol in imaging experiments with brains from line M Thy1-GFP mouse and in immunostaining experiments with antibodies against postsynaptic protein PSD-95 and striatal-specific protein DARPP32.

**Conclusions:**

The original CLARITY protocol was optimized and simplified. Application of the modified CLARITY2 protocol could be useful for a broad range of scientists working in neurobiology and developmental biology.

## Background

Understanding structural organization of the brain is critical for modern neuroscience studies. A number of advanced imaging methods have been developed for studies of brain structure. However, due to light scattering the penetration of light into brain tissue is limited. For confocal microscopy the depth of imaging is limited to 30 micron, for two-photon microscopy it is no more than 600–800 microns [1]. Imaging at such depths also require use of strong excitation power, causing local overheating of the sample. To alleviate the problem of light scattering, recently several procedures have been developed for obtaining optically transparent brain sample for imaging. The simple and fast protocol called See Deep Brain (SeeDB) method was initially published [2]. The SeeDB procedure takes only 1 week, requires minimum reagents and efforts and does not transform the sample. Prepared SeeDB samples are transparent to visible light but not permeable for macromolecules or antibodies. Thus, SeeDB procedure is not compatible with immunostaining. Other methods have been reported that use chemical solvents with high refractive-index to reduce light scattering [3-5]. Similar to SeeDB, these methods are not compatible with immunostaining applications.

The article "Simplified method to perform CLARITY imaging" was published in 2014. Journal: Mol Neurodegener.

The most recently developed method is CLARITY [6]. This method is based on transforming the intact brain tissue to the nanoporous hydrogel formed by cross-linked three-dimensional network of hydrophilic polymers. The lipid phase of the brain is solubilized in detergent and removed by electrophoresis. As a result, optically transparent brain sample is obtained for imaging studies. The nanoporous hydrogel is permeable to the antibodies and other macromolecules, which makes CLARITY compatible with immunostaining applications. However, several steps of published CLARITY protocol [6] are technically difficult. In particular, electrophoretic clearing of the sample is a time consuming and challenging step in the CLARITY procedure.

### New in method

Here we describe a simplified version of the CLARITY procedure (CLARITY2). The initial hydrogel fixation procedure is identical to the original protocol [6]. Following hydrogel fixation, we cut brain tissue in 1–1.5 mm thick coronal slices using vibratome. This additional step enabled us to accelerate and simplify clearing, staining and imaging steps when compared to the original protocol. Using CLARITY2 procedure, we have been able to obtain high quality confocal and two-photon images of neuronal structures from Thy1-GFP transgenic mice [7] and following immunostaining of brain samples with antibodies against synaptic protein PSD-95 and striatal-specific protein DARRP-32.

## Results and discussion

The adult wild type mice (FVB strain) was used to develop the protocol. The mouse brain was obtained and embedded into hydrogel by following previously described protocol [6] without any modifications (see Methods for details). The next step in the published protocol is clearing from lipid/detergent micelles. The original procedure [6] requires use of electrophoretic clearing chamber (ETC.) for the purpose of clearing the sample. This step is technically difficult and numerous variations of ETC. chamber design have been described since initial publication (http://forum.claritytechniques.org). However, based on our own experience and experience of other laboratories (http://forum.claritytechniques.org) the clearing step remains challenging and takes substantial amount of time and effort. We reasoned that clearing whole brain is complicated and slow process, but for most applications it is not necessary to keep whole brain intact. Using vibratome (World Precisions Instruments) we cut the hydrogen-fixed mouse brains to 1–1.5 mm thick coronal slices (Figure 1A). These slices were put into 50 ml conical tubes filled with 10 ml of clearing solution for 7 days (37°C, shaking at 21 rpm, fresh solution changes every 3 days). We discovered that this simple step resulted in efficient clearing of the slices (Figure 1A). In order to speed up clearing procedure standard protein electrophoresis chamber (for example from BioRad) can also be utilized. If electrophoresis chamber is used, then the slices clearing procedure takes 2–3 days when compared to 7 days with passive clearing. The quality of images obtained with passive and electrophoresis-based approach was similar, and we present images from passively cleared samples in this paper.

The article "Simplified method to perform CLARITY imaging" was published in 2014. Journal: Mol Neurodegener.

**Figure 1:** **Simplified CLARITY clearing procedure. (A)** Hydrogel-embedded coronal slices before (bottom) and after (top) passive clearing procedure. **(B)** Coronal slices on microscope cover glass prepared for imaging. **(C)** Confocal images of striatal region co-stained with DARPP32 (green) and PSD-95 (red) antibodies. **(D)** Confocal images of hippocampus region stained with PSD-95 antibodies (red). Scale bar is 150 microns on panels **C**-**D**.

In our pilot experiments the cleared slices were immunostained with mouse monoclonal antibodies against post-synaptic density protein PSD-95 and rabbit monoclonal antibodies against striatal specific protein DARPP32. Original CLARITY procedure required 2 weeks incubation with primary and secondary antibodies to enable sufficient penetration of antibodies into the sample [6]. Coronal slices in our experiments could be efficiently stained after 2 days incubation with primary antibodies and overnight incubation with secondary antibodies. The stained structures were visualized by Alexa-488-conjugated anti-rabbit and Alexa-594-conjugated anti-mouse secondary antibodies. For imaging experiments coronal slices were positioned on microscope slides in PBST solution and covered by a cover slip (Figure 1B). Imaging in flat slices (Figure 1B) did not require use of FocusClear solution needed for image reconstruction at depths more than 2 mm [6]. Using confocal microscope (Thorlabs) equipped with 20x Olympus objectives we have been able to easily visualize the DARRP-32-positive and PSD-95-positive (Figure 1B) structures in the brain samples. The example of striatal region co-stained for PSD-95 (red) and DARPP-32 (green) is shown on Figure 1C. The hippocampal region stained for PSD-95 (red) is shown on Figure 1D. We attempted to compare the quality of images obtained with original [6] and modified procedure, but run into technical difficulties with ETC-clearing step when using original protocol (data not shown). As a result, we have not been able to obtain cleared brain samples using original procedure.

The article "Simplified method to perform CLARITY imaging" was published in 2014. Journal: Mol Neurodegener.

To demonstrate versatility of the modified method we also processed the sections obtained from Thy-GFP mice (line M) brains [7]. In these experiments 1–1.5 mm thick coronal sections from line M mice were passively clarified as described above. The images of GFP-positive hippocampal neurons were collected using confocal microscope equipped with 20x (Figure 2A) or 60x (Figure 2B) Olympus objectives.In the next series of experiments we used anti-PSD95 mouse monoclonal antibodies and Alexa-594-conjugated anti-mouse secondary antibodies to stain coronal sections from line M brains. Obtained confocal images were used for 3D reconstruction of neuronal structures (Figure 3A and B). On these images individual GFP-positive neurons (green) are surrounded by PSD-95-positive synaptic structures (red).

**Figure 2:** **Confocal images of hippocampal neurons from line M Thy1-GFP mouse. (A)** Neuronal structures of hippocampus, 20x objective. Scale bar is 300 microns. **(B)** 3D reconstruction of individual GFP-positive neuron, 60x objective.

**Figure 3:** **Confocal images of striatal and hippocampal neurons from line M Thy1-GFP mouse. (A, B)**. 3D reconstruction of GFP-positive neurons (green) and PSD95 staining (red) is shown. 20x objective was used. Different brain regions are shown on panels **(A)** and **(B)**. Scale bar is 100 microns on panels **A** and **B**.

The results shown on Figures 1, 2 and 3 validate the modified procedure for confocal imaging and immunostaining experiments. Using 20x objectives we have been able to image up to depth of 250 microns using confocal microscopy (Figure 1, 2 and 3). When the samples were imaged with two-photon microscope (Thorlabs, 20x Olympus objective), the depth of penetration was increased up to 1–1.5 mm, that is spanning whole thickness of the slice. The 3D reconstruction of neuronal shapes based on two-photon imaging data is shown for line M GFP-positive neurons on Figure 4 and Additional file 1.

**Figure 4:** **Two-photon imaging of hippocampal neurons from line M Thy1-GFP mouse.** Single frame from 3D neuronal image reconstruction (Additional file 1). 20x objective was used. Scale bar is 150 micron.

The article "Simplified method to perform CLARITY imaging" was published in 2014. Journal: Mol Neurodegener.

In conclusion, here we describe modified and simplified version of CLARITY protocol (CLARITY2). Following imbedding into the hydrogel, the brain samples were cut into 1–1.5 mm thick coronal slices by vibratome. As a result, clearing, immunostaining and imaging procedures have been accelerated and simplified. Clearing could be performed by passive incubation of slices in the clearing solution for 1 week and did not require a special ETC. chamber. Active clearing could be also done with brain slices using standard protein electrophoresis chamber to shorten the clearing procedure to 2–3 days in duration. Antibody staining and imaging steps were also simplified and accelerated when compared to the original protocol. We achieved 250 micron penetration into the thickness of the slice using confocal microscope and have been able to image whole thickness of the slice (1.5 mm) using two-photon microscopy. Imaging in flat slices could be performed on microscope slides and did not require use of expensive FocusClear solution needed for image reconstruction at depths more than 2 mm [6]. We hope that described CLARITY2 procedure will be useful for mapping neuronal circuits in mice brain and for imaging post-mortem human brain samples. When compared to original CLARITY procedure [6] analysis of images obtained using CLARITY2 procedure may require digital “stitching” of images from adjacent coronal sections, but this can be done relatively easily when necessary using image analysis software.

## Methods

### Mice

Wild type FVB/NJ (Stock Number: 001800) or line M mice Tg(Thy1-EGFP)MJrs/J (Stock Number: 007788) [7] were used. Both lines were obtained from the Jackson Laboratory and the breeding colonies were established in the animal facility located in the Laboratory of Molecular Neurodegeneration in St Petersburg State Polytechnical University. All mouse experiments have been performed according to the procedures approved by the local animal control authorities.

### Hydrogel and clearing solutions

Both solutions were prepared by following protocol described in the original article [6]. Briefly, to prepare hydrogel solution combine and mix 40 ml of acrylamide (40%), 10 ml of bis-acrylamide (2%), 1 g of VA-044 initiator (10% wt), 40 ml of 310 PBS, 100 ml of 16% PFA and 210 ml of dH2O. Hydrogel solution is stored at -20°C, all manipulations with hydrogel are performed on ice. For clearing solution combine and mix 123.66 g boric acid, 400 g sodium dodecyl sulphate, and 9 l dH2O. Add dH2O to 10 l and add NaOH until the pH has reached 8.5. This solution can be made, stored and used at room temperature (20°C). To avoid skin contact or inhalation, prepare solutions in a fume hood wearing gloves while preparing both of them.

The article "Simplified method to perform CLARITY imaging" was published in 2014. Journal: Mol Neurodegener.

### Mice perfusion

Thaw the 40 ml of hydrogel at room temperature. Gently mix the content, avoid air bubbles. Keep the tube with hydrogel on ice. Provide animal anesthesia – in our experiments mice were anesthetized with 300 ul of Urethane (250 mg/ml). Transcardially perfuse the mouse with 20 ml of ice-cold solution of hydrogel with perfusion rate of 10 ml per minute. Quickly extract the brain and place it in a conical tube containing remaining 20 ml of hydrogel. Wrap tube in aluminum foil if the sample contains fluorescent substance (such as GFP) to avoid photobleaching. Place the tube in a refrigerator (4°C) for 1–2 days to ensure full penetration of the sample by hydrogel.

### Hydrogel tissue embedding

Tissue embedding was performed according to the protocol described in the original article [6]. Briefly, 50 mL conical tube containing hydrogel-soaked brain sample was positioned to the dessication chamber in a fume hood. The dessication chamber is filled with the nitrogen gas from the tank. Switch the desiccation chamber valve from nitrogen gas flow to the vacuum pump. Keep the vacuum on for 10 minutes, then switch the vacuum off and slowly fill the dessication chamber with the nitrogen gas. Open the dessication chamber and tightly close the top of the sample tube. Minimize exposure of the sample to air as oxygen impedes formation of hydrogel. Submerge the tube in 37°C incubator on the rotator. Incubate for 3 hours or until solution has polymerized. In a fume hood, extract the hydrogel-embedded brain sample from the gel.

### Tissue clearing

Coronal slices (1–1.5 mm in thickness) were cut from hydrogel-embedded brain using World Precisions Instruments vibratome (NVSLM1 Motorized Advance Vibroslice). The slices are numbered, placed in 50 ml plastic tubes and incubated in 10 ml clearing solution for 7–10 days at a temperature of 37C with shaking 21 rpm. Fresh clearing solution was exchanged every 3 days. The clearing of tissue was evaluated by eye. In most experiments 7 days was enough for complete clearing, but for some samples additional 3 days of clearing was needed. The standard Bio-Rad chamber for Western blotting (Mini-Protean Tetra Cell system # 165–8000) could be used to speed up a clearing to 2–3 days in needed. If electrophoretic clearing is used, the chamber is placed to a thermostat at 37°C, and the voltage is set for 12 V. Following passive (7 days) or electrophoretic (2–3 days) clearing the slices are washed from clearing solution in PBST (0.1% Triton X- 100 in PBS) for 2 days. The slices are now clarified.

The article "Simplified method to perform CLARITY imaging" was published in 2014. Journal: Mol Neurodegener.

### Immunochemistry

The cleared brain slices are placed in PBST. The primary antibody is added at 1:1000 dilution for 2 days, then slices are washed with PBST 5 times for 30 minutes. The secondary antibody is added at 1:1000 overnight in PBST, and the slices washed once for 30 min in PBST. The antibodies used in our experiments were: mouse monoclonal anti-PSD-95 (Pierce, MA1-045), rabbit monoclonal anti-DARPP32 (Cell Signaling 19A3), Alexa Fluor488 Goat anti-rabbit (Life Technologies, A-11008), Alexa Fluor594 Goat anti-mouse (Life Technologies, A-11005).

### Imaging

The slices are removed from PBST and put on a glass slide. The slices are covered with the cover glass, which is cemented to the glass slide using plastiline (Figure 1B). The coronal slices are put on the microscope slide in the small drop of liquid (PBST) to avoid drying and to prevent formation of air bubbles. The plastiline is mounted around the sample and the sample is covered with a cover slip. Be very careful to avoid trapped air bubbles. Confocal and 2 –photon imaging systems (ThorLabs) equipped with 20× and 60× Olympus objectives (w.d. 2.0 mm) were used in our imaging experiments. Obtained images were analyzed using Imaris v7.4.2. Software.

## Competing interests

The authors declare that they have no competing interests.

## Authors’ contributions

EP and DA performed the experiments. EP, DA, AB analyzed data. EP, DA, OV and IB designed research. EP, DA, AB, OV, IB wrote the paper and prepare figures for publication. All authors read and approved the final manuscript.

## Authors’ information

Ekaterina Poguzhelskaya at poguzhelskaya@mail.ru is a contact for technical questions on the procedures described in this paper.

## Supplementary Material

Additional file 1 **3D reconstruction of hippocampal neurons form line M Thy1-GFP mice based on two-photon imaging data (20 x objective).** Click here for file
